The article "Efficacy and Safety of Tripterygium Wilfordii Glycoside Tablets Combined with Acitretin Capsules in the Treatment of Moderate to Severe Plaque Psoriasis: A Randomized Controlled Trial" was retracted in 2023. Reasons: signs of a paper mill; compromised peer review; unreliable results or conclusions.

# Efficacy and Safety of Tripterygium Wilfordii Glycoside Tablets Combined with Acitretin Capsules in the Treatment of Moderate to Severe Plaque Psoriasis: A Randomized Controlled Trial

**DOI:** 10.1155/2022/2252500

**Published:** 2022-07-09

**Authors:** Qinghui Fu, Yunjie Zhu, Yiqi Fang, Changbo Dai

**Affiliations:** ^1^Department of Dermatology, Zunyi Hospital of Traditional Chinese Medicine, No. 8, Fenghuang South Road, Honghuagang District, Zunyi City, Guizhou 563099, China; ^2^Department of Nephrology, Suzhou Hospital of Traditional Chinese Medicine, No. 18, Yangsu Road, Canglang New Town, No. 889, Wuzhong West Road, Suzhou, Jiangsu 215009, China; ^3^Department of Hematology, Suzhou Hospital of Traditional Chinese Medicine, No. 18, Yangsu Road, Canglang New Town, No. 889, Wuzhong West Road, Suzhou, Jiangsu 215009, China; ^4^Department of Dermatology, Suzhou TCM Hospital Affiliated to NanJing University of Chinese Medicine, No. 18, Yangsu Road, Canglang New Town, No. 889, Wuzhong West Road, Suzhou, Jiangsu 215009, China

## Abstract

**Objective:**

To probe into the clinical efficacy of tripterygium wilfordii glycoside (TWGs) tablets combined with acitretin capsules in the treatment of patients with moderate to severe plaque psoriasis (MSPP).

**Methods:**

Thirty-six patients with MSPP were collected and divided into three groups, namely, group A (*n* = 12, TWG tablets + acitretin capsules), group B (*n* = 12, compound glycyrrhizin capsules + acitretin capsules), and group C (*n* = 12, acitretin capsules). The general data of the patients was recorded. In addition, a comparison was made before treatment, 4 weeks and 8 weeks after treatment in terms of the clinical efficacy, liver function indicators (alanine aminotransferase (ALT), aspartate transaminase (AST), and creatinine), psoriasis area, and severity index (PASI) scores. The incidence of adverse reactions after treatment and the recurrence rate during two months of follow-up was statistically analyzed.

**Results:**

The therapeutic effect of group A was superior to the other two groups, with obviously more satisfactory results of serum parameters, clinical efficacy and PASI score, and incidence of adverse reactions.

**Conclusions:**

TWGs combined with acitretin had better therapeutic effects and higher safety in the treatment of MSPP.

## 1. Introduction

Psoriasis is an immune-mediated chronic skin disease that affects roughly 125 million people worldwide [1]. Psoriasis is comprised of plaque psoriasis (PP), guttate psoriasis, erythrodermic psoriasis, and pustular psoriasis [2]. Among the four subcategories, PP constitutes the most common variant of psoriasis, accounting for more than 80% of psoriasis cases [3]. It is characterized by the presence of erythematous scaly plaques on the extensor surface as well as on the other frictional areas, such as palms, soles, and nails. The affected areas are typically well defined and usually symmetrical [4], and clinically, psoriasis is classified as mild, moderate, and severe based on the affected area of the patient. To be specific, psoriasis with less than 3% to 5% of affected body surface area is defined as mild one, those with 3% or 5% to 10% as moderate one, and those with more than 10% as severe one [5]. For patients with moderate to severe psoriasis, the main therapy involves phototherapy and drug therapy, but the application of the former has been reduced in clinical practices nowadays. Drug therapy is mainly based on biological agents and oral drugs. Oral drugs have been used to treat moderate to severe PP (MSPP) for many years; however, the therapeutic effect of MSPP is not satisfactory due to multiple drug contraindications. Therefore, new treatment strategies are required to improve the current status.

Acitretin, a synthetic aromatic retinoid as well as an active metabolite of etretinate, has been used in the treatment of severe psoriasis for many years, whose therapeutic potency has long been proven better than that of traditional systemic therapy. Unlike other systemic therapies, acitretin is not an immunosuppressor. Instead, it exerts an antipsoriatic activity to normalize keratinocyte differentiation and proliferation and indirectly modulates the inflammatory response [6]. Common adverse reactions caused by acitretin include xerosis, rhinitis, nail dystrophy, elevated levels of serum triglycerides, and liver enzymes. These side effects are usually reversible after discontinuation of treatment [7]. However, data from recent studies on the efficacy and safety of acitretin are conflicting [8]. Some studies have pointed out the increased frequency of adverse events and abnormalities due to dose-dependent acitretin [7], suggesting that attention should be paid to the clinical use of acitretin dose.

Tripterygium wilfordii glycosides (TWGs) are lipid-soluble mixtures extracted and refined from the roots of Tripterygium wilfordii Hook F, a member of the celastraceae plant. TWGs act to eliminate dampness, disperse swelling, dispel wind, and detoxify [9]. According to modern pharmacological studies, TWGs also show specific anti-inflammatory and immunomodulatory effects [10]. Although the pathogenesis of PP is very complex and has not been fully elucidated, some studies have believed that excessive activation of the adaptive immune system, mainly the change of T helper 17 (Th 17) cell status, may be the core of the pathogenesis of psoriasis [11]. TWGs have been approved for the clinical treatment of patients with rheumatoid arthritis, nephrotic syndrome, ankylosing spondylitis, psoriasis, and systemic lupus erythematosus [12]. In addition, TWGs are able to inhibit IL-17A derived from Th17 cells and improve psoriasis by interrupting the phosphorylation of signal transducer and activator of transcription 3 (STAT3) [13]. Glycyrrhizin alone or combining with TWGs have been reported to have a better therapeutic activity than normal clinical treatment for psoriasis vulgaris [14, 15]. However, whether the combination of acitretin with TWGs or glycyrrhizin could create a more efficient therapy for MSPP is still unknown. Therefore, this study attempts to explore the effects of these combination of the drugs in clinical practice and provide a new therapeutic idea for the treatment of this disease.

## 2. Materials and Methods

### 2.1. Study Subjects

A total of 36 patients with MSPP received treatment in our hospital between January 1, 2018 and June 1, 2021 were collected. They were divided into group A (*n* = 12, TWG tablets + acitretin capsules), group B (*n* = 12, compound glycyrrhizin capsules + acitretin capsules), and group C (*n* = 12, acitretin capsules alone).

Inclusion criteria of the patients who were (1) diagnosed as MSPP by clinical examination, (2) aged over 18 years old, (3) signed an informed consent for this study, (4) with seven points < psoriasis area and severity index (PASI) score < 20 points, (5) without drug treatment and topical medication for skin lesions within 6 months, and (6) with good compliance to ensure effective observation and accurate data throughout the treatment.

Exclusion criteria were the patients (1) who suffered from severe hepatic and kidney function damage, cardiovascular disease, and autoimmune diseases; (2) who had coagulation dysfunction; (3) who were diagnosed with allergic diseases; (4) who had malignant tumors; (5) who were in either pregnancy or lactation period; (6) who contraindicated or withdrawn during the administration; and (7) who had mental illness, severe cognitive impairment, or language problems.

General data of the patients were recorded, including age, gender, body mass index (BMI), serum triglyceride (TG), total cholesterol (TC), high-density lipoprotein cholesterol (HDL-c), low-density lipoprotein cholesterol (LDL-c), white blood cell count (WBC), and platelet levels.

All patients were provided and signed a written informed consent prior to participation. The study protocol was fully compliance with the Declaration of Helsinki and other bioethical principles. This study was approved by the Medical Ethics Committee of Suzhou Hospital of Traditional Chinese Medicine.

### 2.2. Detection of Serum Indicators

Blood was collected from patients and centrifuged at 3500 r/min for 10 min at 4°C. The supernatant was then obtained to measure the levels of alanine aminotransferase (ALT), aspartate transaminase (AST), and creatinine using an BS-280 Automatic Biochemical Analyzer (Mindray, Shanghai, China).

### 2.3. Psoriasis Area and Severity Index (PASI) Score

To calculate PASI scores, the body was divided into four regions, each with corresponding coefficient according to its degree of extension (head = 0.1, upper limbs = 0.2, trunk = 0.3, lower limbs = 0.4). Plaque characteristics (erythema, induration/thickness, and scaling) were scored individually for each area, and then the scores were summed to get the final score. Subsequently, the PASI scores of all patients were assessed by two dermatologists certified by independent committees and eventually averaged. Should any major discordance (greater than 5% difference in calculated PASI score given by the two dermatologists) be spotted, then a dermatologist certified by the third committee would join the discussion of the case and be responsible for confirming the final conclusion.

### 2.4. Statistical Analysis

All data were analyzed with SPSS 26.0 software (IBM-SPSS, Chicago, IL, USA). For measurement data, they were expressed as mean ± standard deviation (SD), and the comparison between the two groups was analyzed by *t*-test. For enumeration data, they were expressed as *n* (%), and statistical analysis was performed using the chi-square test. A value of *p* < 0.05 indicated a statistically significant result.

## 3. Results

### 3.1. General Information

The average age, weight, height, age of onset, course of disease, and location of the skin lesion did not show any significant differences among the three groups, (Table 1) indicating that the three groups of patients were completely comparable.

### 3.2. TWGs Combined with Acitretin Capsules Display Better Efficacy

In the comparison of the biochemical indicators and PASI scores, no significant differences were identified among the three groups in PASI scores, ALT, AST, and creatinine before treatment. Four weeks after treatment, there was no significant difference was spotted as well in the serum biochemical indicators and PASI scores among the three groups. However, eight weeks after treatment, compared with group C, the PASI scores, serum ALT, AST, and creatinine contents, were remarkably lower, in group A and group B (*p* < 0.05). Noteably, the alteration of the indexes was more significant changed in group A (*p* < 0.05; Figures 1(a)–1(d)).

Thus, the results clearly demonstrated that the best liver function parameters and the best therapeutic effect were obtained in group A. With further observation on the skin status, significant improvement was found in group A as well (Figure 1(e)).

In the comparison of the effective rate, four weeks after treatment, two patients recovered, four patients showed significant improvement, and six patients demonstrated symptoms of improvement in group A, indicating that the effective rate of group A reached as far as 100%, which was significantly higher than that in group B (83.33%) and group C (58.33%) (*p* < 0.05). In addition, eight weeks after treatment, the effective rate of the group A was 100% (cured: *n* = 8; significantly effective: *n* = 3; effective: *n* = 1) as well, which was much better than that of group B (91.67%) and group C (66.67%) (*p* < 0.05) (Table 2).

### 3.3. TWGs Combined with Acitretin Capsules Reduced Adverse Reactions and Recurrence in Patients

The adverse reactions of the 36 patients after treatment were statistically analyzed. The results showed that totally 11 patients (30.6%) had adverse reactions, including one patient (8.33%) in group A, two (25.0%) in group B, and seven (58.3%) in group C (Table 3). Thus, the incidence of adverse reactions was significantly lower in the patients of group A than that in groups B or C.

Additionally, during the follow-up lasting two months, no recurrence was recorded in group A and B, while three patients (25.0%) were found in group C four weeks after treatment. Further, eight weeks after treatment, group A still had no cases of recurrence, whereas there were two relapse cases (16.7%) in group B and five relapse cases (41.7%) in group C. Overall, group A had the best effect and the lowest recurrence rate of the adverse reactions among the three groups, while group C had the highest recurrence rate of the adverse reactions (Table 4).

## 4. Discussion

As a condition with complicated etiology, psoriasis results primarily from an abnormal immune response in the skin that is influenced by genetic susceptibility and various environmental stimuli (such as skin trauma, infection, and drug therapy). Early observations suggest that the development of psoriasis is associated with an immune response, resulting in skin lesions with increased amount of inflammatory cells infiltrating [16]. Dysregulation of the inflammatory response is a key cause of psoriasis. Although the mechanism of relieving inflammation in psoriasis remains to be elucidated, a variety of traditional Chinese medicines have been shown to be effective in autoimmune diseases such as TWGs. TWGs can effectively mitigate the serum levels of inflammatory factors in patients with chronic nephritis by inhibiting the production of proinflammatory mediators and regulating the microbial population [17]. Aside from the effects mentioned above, TWGs make contributions to preventing colon shortening and alleviate the histological inflammation of the intestinal mucosa by prohibiting proinflammatory cytokines increase [18]. TWGs also act to attenuate Th17 cell differentiation and enhance Treg differentiation [19]. In this study, we found that TWGs combined with acitretin capsules significantly reduced PASI score and were thus of certain efficacy, indicating that TWGs can significantly boost the efficacy of acitretin and reveal better therapeutic affect than that of the glycyrrhizin+acitretin in MSPP.

For patients with mild psoriasis, topical agents remain the primary therapy, including topical corticosteroids, vitamin D analogues, calcineurin inhibitors, and keratolytics agents [20]. For MSPP, oral drugs or biological agents are required. Oral medications include methotrexate, apremilast, acitretin, and cyclosporine. Although all of those are generally less effective than biological agents except cyclosporine, biological agents may induce more side effects and adverse effects [21]. Therefore, oral therapeutic drugs remain the dominant drugs in clinical practice. Unfortunately, oral drugs, including acitretin, have also been found to result in hepatotoxicity in patients [22]. Rapid control of MSPP usually requires high-dose acitretin (0.5-1 mg/kg/day) in the acute phase [23]. Acitretin used in this study was less than 0.5 mg/kg/day, and the results showed that TWGs combined with acitretin capsule significantly reduced liver injury compared with the other two treatment methods. Previous studies have shown that acitretin inhibits Th17 cell differentiation through the retinoic acid-related receptor ROR*γ*t, a key transcription factor for Th17 cell development [24]. Zhang et al. came to the conclusion that TWGs inhibited Th17 cell differentiation by inhibiting RORC and STAT3 expression, while promoting Treg cell differentiation by enhancing the Foxp3 expression in CD4^+^ T cells [25]. Besides, TWGs can also act on HIF1*α* to regulate the balance of Th17/Treg [26]. In this study, the combination of TWGs and acitretin capsules achieved best efficacy with lowest recurrence rate, which may be ascribed to the enhanced regulatory effect of acitretin on immune response by TWGs. To sum up, our study proves that compared with glycyrrhizin+acitretin and acitretin alone treatment methods, TWGs combined with acitretin capsules exert a more remarkable effect in patients with MSPP, with a high effective rate and low incidence of side effects. Therefore, this combined therapy should be promoted in clinical practice.

## 5. Conclusions

Collectively, TWGs combined with acitretin capsules can effectively treat MSPP, improve the clinical symptoms of patients, and minimize the recurrence rate and adverse reactions. Therefore, this treatment is worth popularizing in clinical application. Nonetheless, this study still has some limitations, such as inadequate samples and the lack of various regional backgrounds of the patients included. Obtaining more comprehensive data for its clinical use requires further exploration of the therapeutic effects of this method.

## Figures and Tables

**Figure 1:** Comparison of treatment efficacy among the three groups. Psoriasis area and severity index (PASI) score (a), serum alanine aminotransferase (ALT) level (b), serum aspartate transaminase (AST) (c), and serum creatinine (d) level were detected in the patients of the group A (blue), group B (green), and group C (red). (e) Representative images showed the area of skin erythema before and after treatment with WTGs+acitretin (group A). ∗∗*p* < 0.01 vs. group C; ##*p* < 0.01 vs. group B. Group A, TWG tablets + acitretin capsules; Group B, compound glycyrrhizin capsules + acitretin capsules; Group C, acitretin capsules alone.

**Table 1:** General information of the patients in the three groups.

	Group A	Group B	Group C	*p*
Age (years)	36.17 ± 5.29	36.50 ± 3.83	36.00 ± 4.31	0.963
Gender				0.717
Male	7	6	5	
Female	5	6	7	
Height (cm)	170.67 ± 8.30	170.33 ± 10.33	170.92 ± 9.98	0.989
Weight (kg)	69.17 ± 15.57	68.00 ± 16.64	68.33 ± 13.19	0.981
Age of onset (years)	34.00 ± 4.65	33.83 ± 3.38	33.92 ± 4.23	0.995
Course of disease (years)	2.16 ± 1.34	2.67 ± 1.56	2.08 ± 1.00	0.509
Location of skin lesion				0.945
Head and neck	2	1	1	
Trunk	8	8	8	
Limb	2	3	3	
Extent coverage by skin lesion				0.929
<30%	1	1	1	
31%-50%	5	4	6	
51%-70%	3	5	4	
>71%	3	2	1	
Complications				0.793
Related to psoriasis	10	11	10	
Not related to psoriasis	2	1	2	
TG (mmol\L)	1.34 ± 0.17	1.34 ± 0.06	1.35 ± 0.11	0.985
TC (mmol\L)	4.53 ± 0.26	4.56 ± 0.35	4.55 ± 0.29	0.962
HDL-c (mmol\L)	1.32 ± 0.11	1.33 ± 0.17	1.33 ± 0.15	0.993
LDL-c (mmol\L)	2.75 ± 0.13	2.75 ± 0.21	2.74 ± 0.26	0.969
WBC (×10^9^/L)	7.27 ± 0.24	7.28 ± 0.15	7.28 ± 0.15	0.991
Platelet (×10^9^/L)	229.17 ± 20.74	229.50 ± 21.55	228.93 ± 14.65	0.997

Data was mean ± SD or *n*. Group A, TWG tablets + acitretin capsules; Group B, compound glycyrrhizin capsules + acitretin capsules; Group C, acitretin capsules alone. TG: triglyceride; TC: total cholesterol; HDL-c: high-density lipoprotein cholesterol; LDL-c: low-density lipoprotein cholesterol; WBC: white blood cell count.

**Table 2:** Comparison of clinical efficacy among three groups.

	Cured	Significantly effective	Effective	Noneffective	Effective rate (%)	*p*
Four weeks after treatment						
Group A	2	4	6	0	100.00	0.034
Group B	0	5	5	2	83.33	
Group C	0	4	3	5	58.33	
Eight weeks after treatment						
Group A	8	3	1	0	100.00	0.049
Group B	4	6	1	1	91.67	
Group C	2	4	1	4	66.67	

**Table 3:** Comparison of adverse reactions among three groups.

	Group A	Group B	Group C	*p*
Dry mouth	0	1	1	0.589
Loss of appetite	1	0	0	0.358
Abdominal pain	0	0	1	0.358
Nausea and vomiting	0	1	3	0.140
Elevated urea ammonia	0	0	1	0.358
Menstrual disorder	0	0	1	0.358
Total	1	2	7	0.026

**Table 4:** Comparison of recurrence rate among three groups.

	Group A	Group B	Group C	*p*
Four weeks after treatment	0	0	3	0.038
Eight weeks after treatment	0	2	5	0.034

## Data Availability

The data used to support the findings of this study are available from the corresponding author upon request.
